# Clinical Application of a Safe Blood Sampling Device with an Indwelling Needle

**DOI:** 10.1155/2022/6362905

**Published:** 2022-09-01

**Authors:** Yeqin Deng, Zhengbing Lv, Yue Cheng, Annuo Liu, Zhengling Huang

**Affiliations:** ^1^Anhui Maternal and Child Health Hospital, Anhui Medical University, Hefei, Anhui, China; ^2^Zhejiang Sci-Tech University, Hangzhou, Zhejiang, China; ^3^School of Nursing, Anhui Medical University, Hefei, Anhui, China

## Abstract

**Background:**

The traditional indwelling needle catheter is hard and can only complete one puncture at a time. The safety and indwelling needle catheter is soft, with a large lumen, with high success rate of blood collection, and one puncture completes two operations, so it is of important value and significance to study the new safety and indwelling needle. To explore the clinical utility of a novel blood collection device with indwelling needle for blood collection among pediatric patients.

**Methods:**

A total of 300 children who were admitted to the children's hospital from March to June 2020 were selected and randomly divided into the control group (148) and the observation group (152). The control group received venipuncture using regular needles for infusion and blood collection. For the observation group, a modified indwelling needle device was used for the procedures. Comparisons were made between the two devices in five aspects: blood sample quality, operation time, needlestick incidence, related complications, and patient satisfaction.

**Results:**

There was no significant difference in coagulation rate between the two groups, but slightly lower overall hemolysis incidence in the observation group. The unqualified rate of blood specimens collected in the observation group was 10.0% lower than that in the control group (*P* < 0.05). Shorter operation time, lower incidence of needlestick injuries, and improved satisfaction were observed in the group using the novel blood collection device.

**Conclusions:**

This modified blood collection device is superior to the regular venipuncture needle, in terms of safety, efficiency, and patient satisfaction; thus, it has potential for broad clinical applications for infusion and blood collection.

## 1. Introduction

Intravenous (IV) infusion and blood sampling are routine and important procedures for sick children for timely diagnosis and effective treatment, and most hospitalized children need vessel puncture and blood sampling. An intravenous catheter has been most commonly used clinically as a blood sampling device, allowing long venous access with simple procedure [1]. Studies show that the incidence of needlestick injury among nurses in China was 57.3% [2]; the incidence among intern nurses is even higher, about 60.8% [3]. Safety needles can be selected to effectively avoid such accidents [4, 5]. Traditional blood sampling devices need to press open the catheter valve inward to facilitate inserting a syringe into the valve in order to draw blood. The blood sample in the syringe is then injected into the sample collection tube. Connecting a syringe to the catheter valve for blood collection is cumbersome and typically involves multiple steps. It also has many disadvantages such as repeated disconnection, difficult to control blood volume, easy infection, and blood clotting [6]. When collecting blood samples from children using the IV catheter, it is easier to make mistakes and inflict needlestick injuries since they are often uncooperative, restless, and crying [7].

To this end, we have developed a novel blood sampling device that is more convenient and simple-to-operate and reduces the possibility of clinical complications. In this paper, the safe and traditional indwelling needle design has a thinner needle tube, a softer catheter, and a larger lumen and greatly improved the success rate of blood collection, and one puncture can complete two tasks. We evaluate the safety and utility of this blood collection device among pediatric patients for infusion and blood sampling procedures in contrast with regular intravenous catheters.

## 2. Design of the Blood Collection Device

A common intravenous catheter was used for a regular blood collection procedure, which is composed of a 22-24G needle at the top connected with a 5 mL syringe, plus a blood drawing syringe with a heparin cap connected with a vacuum collection tube (Figure 1). The details of new design are shown in Figure 2, comprised of a negative pressure large-diameter tube (part 1) attached at the end that can hold and protect the puncture needle (part 2), the connecting soft tubing to the needle (part 3), the puncture needle sheath (part 4), and a threaded adapter (part 5) at the other end suitable for Y type or non-Y type indwelling needle connection. Type Y is an indwelling needle with two exits, usually with an extension tube: one outlet for injection and one with a heparin cap; non-Y type is handling indwelling needles other than Y type and the male (part 6) and female buckle (part 7) at the exterior of the soft tubing. The assembled device with all parts is shown in Figure 3. This new design is more efficient and safer for clinical tasks of blood collection and infusion for pediatric patients who often require both procedures and suffer repeated needle punctures, as both procedures can be achieved in a one-time needle puncture. To avoid contamination of saline or anticoagulant in collected blood sample, a single or multiple blood collections using this device would be conducted before infusion treatment, e.g., blood collection followed by infusion.

## 3. Results

A total of 300 children with the age of 7 years or younger admitted to our hospital from March to June 2020 were selected and randomly divided into a control group (*n* = 148) and an observation group (*n* = 152). The control group consisted of 78 males and 70 females, with an average age of 4.5 ± 2.13 years; clinical manifestations include 74 upper respiratory tract infections, 26 diarrhea, 33 pneumonia, and 15 other diseases. The average age for the observation group was 4.0 ± 2.21 years, which consisted of 82 males and 70 females, with clinical diagnosis of 73 upper respiratory tract infections, 28 diarrheas, 32 pneumonias, and 19 other diseases. There is no statistical difference between the two groups in terms of age, sex, and clinical disease categories (*P* > 0.05).

A total of 750 tubes of blood samples were collected, 350 tubes in the control group (148 patients) and 400 tubes in the observation group (152 patients). The overall hemolysis rate in the observation group was lower than that of the control group, with statistically significant difference (*P* < 0.05), The hemolysis rate generally has no normal range, but the normal value of the hemolysis index is 1 : 64. If the hemolysis index test result is greater than 1 : 64, the probability of hemolysis is very high as shown in Table 1.

The coagulation rate of the control group was 4.3% (10/230), while that of the observation group was 5.5% (15/275), statistically not significant between the two (*P* > 0.05).

In the comparison of the unqualified rate of specimen collection between the two groups, the unqualified rate of blood specimens in the observation group was 1.3% (5/400), which was lower than 9.4% (33/350) in the control group, and the difference between the two groups was statistically significant (*P* < 0.05).

The blood collection time in the observation group was significantly shorter than that in the control group (*P* < 0.05), and the incidence of needlestick injury was also significantly reduced (*P* < 0.05), as shown in Table 2.

The incidence of complications and patient satisfactions between the two groups were also compared. The incidence of complications associated with the use of new blood collection device in the observation group was significantly lower than that in the control group (*P* < 0.05), and similarly, the rate of patient satisfaction was significantly higher in the observation group (Table 3).

## 4. Discussion

The most common method of blood collection in hospitals or clinics is to use disposable blood collection needle, which requires arterial or venous puncture separately [8]. In order to reduce the number of puncture, an indwelling needle is commonly used in a clinic or hospital for sick children for dual purposes of blood collection and infusion treatment [9]. However, the traditional indwelling needle technique needs connection and disconnection of the needle to allow the syringe to be inserted into the sample collection tube for blood collection. This operation is repetitive and complicated and requiring the right force from both hands to insert the needle into or withdraw from the tube, which may affect the stability of the needle in the vein at the other end [9]. This procedure is especially difficult when performed on children who are often crying and moving, with minimum cooperation, thus more likely causing operational errors or high risk of needlestick injuries [10].

Our design of safe intravenous blood collection device has several features with advantages in clinical practical use over regular blood sampling device. First, the needle-free threaded adapter can reduce the number of punctures and lower the incidence of needle injury of medical staff. Second, the negative pressure tube prevents the puncture needle from hurting the medical staff and provides a safer and sterile operation area. Third, the sheath surrounding puncture needle prevents the puncture needle from air contamination and also reduces the chance of needlestick injury to the medical staff. Finally, the male and female adhesive buckle is simple and convenient, which is used to stop blood flow in the tubing during blood draw when the two adhesive pieces mate, not only avoiding damage to the soft tubing but also improving the efficiency of blood collection. In addition, strict disinfection procedures and catheter flushing were performed to avoid contamination. More importantly, the newly designed blood sampling device has a low cost of about half a US dollar, 2-3 fold cheaper than the price of similar device in China, thus saving a large amount of expenses for hospitals and testing labs if broadly used.

The overall hemolysis rate in observation group is a bit lower than that in the control group. Indeed, children are often uncooperative for a venipuncture at the second time due to fear of needle and thus more difficult to puncture and prone to hemolysis [11]. The chance of hemolysis can be reduced by some methods, such as collecting blood from the indwelling catheter in the anterior elbow area [12].

In the observation group, the percentage of unqualified blood samples collected using the new device was reduced, and the operation time was shortened more than one minute relative to the control group. Insufficient blood is one of the reasons for unqualified blood samples due to the complexity of this operation for pediatric patients [13]. Our design simplified the tasks of blood collection and infusion into a single operation that is convenient and fast so as to improve the efficiency of first aid in health settings.

Our data suggest that the incidence of needlestick injury and complications decreased among the group using the new blood collection device, and the patients' satisfaction also improved. This innovative device has combined the multiple clinical tasks of blood collection, infusion, and intravenous indwelling function into one simple operation, which improve the efficiency of blood sampling and reduce operation time. In the process of blood collection, it also reduces the risk of infection and needlestick injury.

This study has several limitations. First, the sample size in the study cohort is limited, so a larger scale study for comprehensive evaluation of this device in children might be needed. Second, this device was not evaluated in adult patient groups because the study was conducted in children's hospitals. Lastly, the length of time for a needle indwelling in the vein or types of medication used in infusion was not included as confounding factors when identifying complications among the two study groups.

## 5. Conclusions

In summary, this safety blood collection device can be connected easily with different types of indwelling needles using the threaded adaptor, simple to operate and no need of being disconnected repeatedly. It overcomes the shortcoming of the traditional IV indwelling needle in China that serves a single purpose of infusion. One needle puncture in pediatric patients is enough for multiple blood drawings and infusions, which effectively reduce the operation time and the incidence of needlestick injury and also save significant cost for hospitals and other health settings. Of course, this new device should be applicable in adult patients for the same procedures and worthy of further investigation in the future.

## 6. Methods

### 6.1. Study Groups

All experimental studies were carried out in accordance with Anhui Medical University clinical study guideline and regulations. All experimental protocols and study design were reviewed and approved by the Anhui Medical University review board. Informed consent was obtained from either parent or legal guardian of children in the study cohorts.

A total of 300 children admitted to our hospital from March to June 2020 were selected and randomly divided into a control group (odd number in the last digit of patients' admission number) and an observation group (even number in the patients' last digit of admission number), with 148 as the control group and 152 as the observation group. The clinical operation of blood collection was performed by pediatric nurses with standardized training and extensive experience according to the clinical operation standards. The following are the inclusion criteria: (1) those who need to receive both intravenous infusion and venous blood sampling on the day of admission, (2) less than or equal to 7 years old, and (3) the guardian of the child agreeing to participate and sign an informed consent. The exclusion criteria include (1) neonatal hemolysis, (2) patients with skin burns, and (3) children with hypercoagulable state.

### 6.2. Comparisons of Efficiency, Safety, and Complications Associated with the Use of Two Different Blood Sampling Devices

The hemolysis rate and coagulation rate of the samples and percentage of unqualified samples were compared between the two groups. Two professional inspectors independently evaluated the quality of blood collection samples including hemolysis and coagulation. The hemolysis rate was calculated based on the number of hemolytic tubes divided by the number of total tubes. The coagulation rate (%) is the ratio of the coagulation tubes out of total tubes. To meet the clinical blood collection standard, the sample collection volume must be between 2.2 and 3.2 mL for blood coagulation tube, 1.5-1.7 mL for blood sedimentation tube, 3-5 mL for drying tube and heparin tube, and 1-3 mL for EDTA tube. Complications include tube blockage, tube detached, and liquid leakage. The rate of total complications is equal to the sum of all complication occurrences divided by the number of total patients.

The time spent for the blood sampling was determined using a stopwatch from the beginning of skin disinfection to blood collection and to IV infusion. The incidence of needlestick injury and related complications were recorded. The patient satisfaction questionnaire was designed with reference to Kantartjis et al.'s literature [14], comprising of four aspects: nurse's blood collection technology, blood collection time, patient's cooperation, and patients' knowledge about blood sampling via education, with a total score of 100 points. The parents or guardian of the patient would answer the questionnaire if a patient was too young and unable to. A score of ≥90 was considered satisfactory, 70-89 was considered basically satisfied, and <70 was considered dissatisfied. The rate of patient satisfaction (%) = (satisfaction + basic satisfaction)/total number of patients × 100%.

### 6.3. Statistical Analysis

A *t*-test was used to compare the numerical values between two groups, while chi square value (*X*^2^) test used for percentage comparison between groups. The statistical calculation was performed using SPSS23.0 software, with *P* < 0.05 being considered statistically significant.

## Figures and Tables

**Figure 1:** Regular blood collection catheter with a syringe attached.

**Figure 2:** The structural view of the new blood collection device.

**Figure 3:** The outline view of the new device after assembly.

**Table 1:** Comparison of blood specimens of two study groups.

Group	EDTA tube (%)	Dry tube (%)	Blood clotting tube (%)	Heparin tube (%)	Erythrocyte sedimentation tube (%)	Overall hemolysis rate (%)
Control	15/115 (13%)	20/120 (16.7%)	10/50 (20%)	5/55 (9.1%)	1/10 (10%)	51/350 (14.6%)
Observation	15/130 (11.5%)	10/125 (8%)	5/65 (7.7%)	5/70 (7.1%)	0/10 (0)	35/400 (8.6%)
*X* ^2^	0.000	3.346	2.871	0.001	0.000	4.935
*P* value	1.000	0.067	0.090	0.971	1.000	0.026

**Table 2:** Comparison of blood collection time and needlestick injury rate between the two study groups.

Group	Number of blood specimens	Operation time (minutes)	Needle stick injury rate (%)
Control group	350	6.2 ± 1.3	32 (9.1%)
Observation group	400	4.7 ± 1.1	6 (1.5%)
*X* ^2^		5.624	22.669
*P* value		<0.05	<0.05

**Table 3:** Comparison of incidence of complications and patient satisfaction between the two groups.

Group	Number of patients	Tube blockage (%)	Tube detached (%)	Liquid leakage (%)	Total complications (%)	Satisfactory rate (%)
Control group	148	5 (3.3%)	9 (6.1%)	19 (12.8%)	33 (22.3%)	118 (79.7%)
Observation group	152	2 (1.3%)	5 (3.3%)	5 (3.3%)	12 (7.9%)	150 (98.6%)
*X* ^2^					12.2	28.3
*P* value					<0.05	<0.05

## Data Availability

The datasets used and/or analysed during the current study are available from the corresponding authors on reasonable request.
